# Topological analysis of carbon and boron nitride nanotubes

This article has been retracted.

**DOI:** 10.1038/s41598-020-58372-1

**Published:** 2020-01-30

**Authors:** Awais Yousaf, Hanan Alolaiyan, Muhammad Nadeem, Abdul Razaq

**Affiliations:** 1 Department of Mathematics, The Islamia University of Bahawalpur, Bahawalpur, 63100 Pakistan; 2 Department of Mathematics, King Saud University, Riyadh, 11362 Kingdom of Saudi Arabia; 3 Department of Mathematics, University of Education Lahore, Jauharabad, 41200 Pakistan

**Keywords:** Computational chemistry, Computational science

## Abstract

Graph theoretical concepts are broadly used in several fields to examine and model various applications. In computational chemistry, the characteristics of a molecular compound can be assessed with the help of a numerical value, known as a topological index. Topological indices are extensively used to study the molecular mechanics in QSAR and QSPR modeling. In this study, we have developed the closed formulae to estimate ABC, ABC_4_, GA, and GA_5_ topological indices for the graphical structures of boron nitride and carbon nanotube.

## Introduction

Graph theory has been used in almost every field of study. A branch of graph theory that deals with the study of molecular compounds in terms of a simple connected planar graph is known as chemical graph theory. The compound’s atoms are the vertices of graph, where the edges represent the bonds between the atoms. The number of edges associated with a vertex of the graph is called the degree of the vertex; on the other hand, in the chemical graph theory, the degree of a vertex is the valency of the atom. Therefore, the algebraist uses Graph Theory as a tool to understand the structure of a molecular compound. Graph theory is also very effective in studying the structural properties of chemical compounds in quantum chemistry. A numerical quantity called topological index can be used to study the properties of a chemical compound. Some of the graph-related topological indices are based on polynomial, distance, and degree. The Geometric-arithmetic (GA) and Atom-bond connectivity (ABC) are the most studied topological indices and play a dynamic role in characterization of a molecular compound. Over the last five decades, several researchers have been focusing in this area of graph theory^1–7^. H. Wiener introduced the topological index and named it the path number and later the Wiener index^8^. In^1^ S. Hayat and co-authors studied several topological indices based on the degree of vertices for certain graph structures. Imran *et al*. studied the structural properties of graph and developed closed formulae of ABC, ABC_4_, ABC_5_, GA, GA_4_ and GA_5_ indices for sierpinski networks^7^. M. Darafsheh in^9^ determined the Wiener, Padmakar-Ivan and Szeged indices through various technique. Further in^10^ A. Ayesha and A. Alameri examined numerous indices such as; Wiener index, Wiener-type invariants, Hyper-Wiener index, Wiener polarity index, Schultz and modified Schultz indices for mk-graph. Wei Gao and co-authors discussed topological indices for the structures of the cyclo alkane’s family based on the graph’s eccentricity^11^. More information on topological indices and chemical structures of various graphs is available in the literature and suggested for readers^12–19^.

Let $G=(V(G),E(G))$ be a simply connected planner graph, where $\,V(G)$, is the vertex set and $E(G)$, is the set of edges of graph *G*. For any vertex, $x\in V(G)$ then, the set $NG(x)\,=\{y\in V(G)/xy\in E(G)\}$ is called open neighborhood of *x*.

$$Sx=\sum _{y\in {N}_{G}(x)}dy.$$

where ${d}_{y}$ denotes the degree of vertex $y$ and ${s}_{x}$ is the sum of the degrees of all open neighborhoods of $\,x$.

The history of some degree-based topological indices is discussed here; Estrada *et al*.^20^ described the degree-based topological index named the atom-bond connectivity index (ABC). That is,

$$ABC(G)=\sum _{xy\in E(G)}\sqrt{\frac{dx+dy-2}{dxdy}}$$

In^21^, Ghorbani with co-authors gave the closed formulae to compute the fourth version of atom-bond connectivity index ($AB{C}_{4}$). The relation to evaluate the $AB{C}_{4}$ index in terms of sum of degrees of neighboring vertices is;

$$AB{C}_{4}(G)=\sum _{xy\in E(G)}\sqrt{\frac{{s}_{x}+{s}_{y}-2}{{s}_{x}{s}_{y}}}$$

Damir Vukičević and Boris Furtula formulated degree based Geometric-arithmetic index (GA) in^2^ and is defined as;

$$GA(G)=\sum _{xy\in E(G)}\frac{2\sqrt{dxdy}}{dx+dy}$$

In^22^, utilizing the concept of Geometric-arithmetic index (GA), A. Graovac and M. Ghorbani defined the fifth version of Geometric-arithmetic index ($G{A}_{5}$) based on the sum of degrees of neighboring vertices. The fifth version of Geometric-arithmetic index ($G{A}_{5}$) is given as;

$$G{A}_{5}(G)=\sum _{xy\in E(G)}\frac{2\sqrt{{s}_{x}{s}_{y}}}{{s}_{x}+{s}_{y}}$$

For more information see^23–27^.

### Hexagonal boron nitride graph

The hexagonal boron nitride graph is a simple connected planner graph. The horizontal and vertical rings of the hexagonal boron nitride graph are shown in Fig. 1. If *n* denotes the number of horizontal rings, then the total number of rings will be *n* × *n*. The order of the Graph $O|G|$, shown in Fig. 2, is $2{n}^{2}+4n$, and the size $E|G|$ of the graph is, $3{n}^{2}+4n-1$. The name used to symbolize boron nitride is BN. The 2D covalent structure of the boron nitride graph has two types: cubic and hexagonal. In present study, we are considering the graph of hexagonal boron nitride. The melting point of boron nitride is below the pressure at, $\,-{3000}^{^\circ }{\boldsymbol{C}}$’ which shows great thermal stability of boron nitride. The atoms of boron and nitrogen are connected alternatively in the structure of boron nitride and form a hexagonal structure. In the hexagonal network, equal numbers of boron and nitrogen atoms are involved in the formation of hexagons. The bond length between the atoms is, 0.145 nm B-N-B angle, or N-B-N is 120°. The structure of the hexagonal BN is single layered and found in nanotubes.

**Figure 1:** 3 × 3, hexagonal boron nitride graph.

**Figure 2:** $\,n\times n$, hexagonal boron nitride graph.

### Carbon nanotubes graph

The carbon nanotube graph $(CNT)$ is a simple connected planner graph shown in Figs. 3 and 4. The carbon nanotube has two sets of rings, that is; vertical and horizontal. The one set contains $n$ vertical rings and the other set contains, $n-1$ horizontal rings. The carbon nanotube graph shown in Fig. 3, has $4{n}^{2}+4n-1$ number of vertices, and $6{n}^{2}+3n-2,\,$number of edges. The term CNT is used to describe the structure of carbon nanotubes. Most of the carbon nanotubes have diameter close to 1 nm and length of the bond between carbons-carbon atoms and angle between the atoms depends upon the structure of the carbon nanotubes. In this paper, we consider the $\,n\times n$, ($m=n$) rectangular section of the carbon nanotube graph for all $n\ge 2$.

**Figure 3:** Graph of carbon nanotubes.

**Figure 4:** Graph of carbon nanotubes with $n=3$.

**Theorem 1.1**. For, $n\ge 2$ the $ABC$ and $GA\,$indices for the network of hexagonal boron nitride are;

i. $$ABC(BN)=\sqrt{3}{n}^{2}-4(\frac{1}{\sqrt{3}}+\sqrt{2})n+(\frac{1}{\sqrt{3}}-5\sqrt{2})$$
ii. $$GA(BN)=3{n}^{2}-4(1-\frac{4\sqrt{6}}{7})n+7$$

**Proof**: The hexagonal boron nitride graph presented in Fig. 2 has three sorts of edges regarding the degrees of vertices. The edge segment of the boron nitride graph on the premise of degrees of vertices are shown in Table 1 underneath:

i. The ABC index of a graph G is defined as;
  $$ABC(G)=\sum _{xy\in E(G)}\sqrt{\frac{dx+dy-2}{dxdy}}$$
  Hence, we obtained the following result using the values of Table 1 and simplifying it.
  $$ABC(BN)=\sqrt{3}{n}^{2}-4\left(\frac{1}{\sqrt{3}}+\sqrt{2}\right)n+\left(\frac{1}{\sqrt{3}}-5\sqrt{2}\right)$$
ii. The geometric-arithmetic index (GA) is defined as:

$$GA(G)=\sum _{{\rm{xy}}\in {\rm{E}}({\rm{G}})}\frac{2\sqrt{{\rm{dxdy}}}}{{\rm{dx}}+{\rm{dy}}}$$

**Table 1:** Edge segment of BN graph on the premise of degree of vertices.

(*d*_*x*_, *d*_*y*_)	Number of edges
(2, 2)	6
(2, 3)	8(*n*−2)
(3, 3)	(*n*−1)(3*n*−1)

We obtained the following result using the values of Table 1 in the above equation.

$$GA(BN)=3{n}^{2}-4(1-\frac{4\sqrt{6}}{7})n+7$$

**Theorem 1.2**. The $\,AB{C}_{4}$ and $G{A}_{5}\,indices\,$of hexagonal boron nitride graph for, $n\ge 2$ are,

$${\rm{i}}.\,AB{C}_{4}(BN)=\frac{4}{3}{n}^{2}+4\left(\frac{21\sqrt{2}+10}{63}\right)n+\left(2\sqrt{\frac{7}{5}}-8\sqrt{\frac{22}{21}}+8\sqrt{\frac{2}{7}}+\frac{20}{9}\right)$$

$$\mathrm{ii}.\,G{A}_{5}(BN)=3{n}^{2}+\left(\frac{16\sqrt{42}}{13}+\frac{3\sqrt{7}}{2}-8\right)n-\left(\frac{32\sqrt{42}}{13}-\frac{4\sqrt{35}}{3}+\frac{4\sqrt{7}}{2}-\frac{16\sqrt{5}}{9}-7\right)$$

**Proof:** The hexagonal boron nitride graph has six types of edges based on the sum of the degrees of neighborhood. This form of edge partition shown in Table 2 below:

i. The fourth version of ABC index is defined as
  $$AB{C}_{4}(G)=\sum _{xy\in E(G)}\sqrt{\frac{{s}_{x}+{s}_{y}-2}{{s}_{x}{s}_{y}}}$$
  Thus, we have calculated $AB{C}_{4}$ index of hexagonal boron nitride graph, using the values of Table 2 in the above equation;
  $$AB{C}_{4}(BN)=\frac{4}{3}{n}^{2}+4\left(\frac{21\sqrt{2}+10}{63}\right)n+\left(2\sqrt{\frac{7}{5}}-8\sqrt{\frac{22}{21}}+8\sqrt{\frac{2}{7}}+\frac{20}{9}\right)$$
ii. The fifth version of geometry index is defined as;

$$G{A}_{5}(G)=\sum _{xy\in E(G)}\frac{2\sqrt{{s}_{x}{s}_{y}}}{{s}_{x}+{s}_{y}}$$

**Table 2:** Edge partition of BN graph based on the sum of the degrees of neighborhood vertices.

(*s*_*x*_, *s*_*y*_)	Number of edges
(4, 5)	$$4$$
(5, 5)	$$2$$
(5, 7)	$$8$$
(6, 7)	$$8(n-2)$$
(7, 9)	$$4(n-1)$$
(9, 9)	(*n* - 1)(3*n* - 5)

Now, we calculate $G{A}_{5}$ index of hexagonal boron nitride graph, by substituting the values of Table 2 in above expression $G{A}_{5}(G)$. It becomes as follows through easy computations.

$$G{A}_{5}(BN)=3{n}^{2}+\left(\frac{16\sqrt{42}}{13}+\frac{3\sqrt{7}}{2}-8\right)n-\left(\frac{32\sqrt{42}}{13}-\frac{4\sqrt{35}}{3}+\frac{4\sqrt{7}}{2}-\frac{16\sqrt{5}}{9}-7\right)$$

**Theorem 1.3**. For the carbon nanotube (CNT) graph for $\,n\ge 2$, the $ABC\,and\,GA\,indices$ are;

$${\rm{i}}.\,ABC(CNT)=4{n}^{2}+\left(5\sqrt{2}-\frac{14}{3}\right)n-\sqrt{2}$$

$${\rm{ii}}.\,GA(CNT)=6{n}^{2}-\left(\frac{25-16\sqrt{6}}{5}\right)n+\left(4-\frac{12\sqrt{6}}{5}\right)$$

**Proof:** The carbon nanotube (CNT) graph is shown in Fig. 2. The CNT graph has three types of edges in terms of degree of vertices. This sort of edge partition presented below in Table 3.

i. The ABC index of a graph G is defined as;
  $$ABC(G)=\sum _{xy\in E(G)}\sqrt{\frac{dx+dy-2}{dxdy}}$$
  Hence, the index $ABC(CNT)$. evolved through the values of Table 3 and the above relation $ABC(G)$, That is;
  $$ABC(CNT)=4{n}^{2}+\left(5\sqrt{2}-\frac{14}{3}\right)n-\sqrt{2}$$
ii. The geometric-arithmetic index (GA) is defined as:

$$GA(G)=\sum _{xy\in E(G)}\frac{2\sqrt{dxdy}}{dx+dy}$$

**Table 3:** Edge partition of CNT graph based on degree of vertices.

(*d*_*x*_, *d*_*y*_)	Number of edges
(2, 2)	$$2n+4$$
(2, 3)	$$8n-6$$
(3, 3)	$$6{n}^{2}-7n$$

Therefore, the required geometric-arithmetic index calculated through the values of Table 3 and simplifying the above expression. We get,

$$GA(CNT)=6{n}^{2}-\left(\frac{25-16\sqrt{6}}{5}\right)n+\left(4-\frac{12\sqrt{6}}{5}\right)$$

**Theorem 1.4**. The $AB{C}_{4}$ and $G{A}_{5}\,indices\,$of carbon nanotube graph for $n\ge 3$ are;

i. $$AB{C}_{4}(CNT)=\frac{8}{3}{n}^{2}+\left(\frac{1}{2}\sqrt{\frac{7}{2}}+\sqrt{\frac{10}{3}}+\frac{22\sqrt{2}}{15}+\frac{2\sqrt{22}}{21}-\frac{14}{3}\right)n-\left(\frac{1}{2}\sqrt{\frac{7}{2}}+\sqrt{\frac{10}{3}}\,+\frac{\sqrt{2}}{3}-2\sqrt{\frac{7}{5}}+5\sqrt{\frac{22}{21}}-8\sqrt{\frac{2}{7}}+\frac{10}{9}\right)$$
ii. $$G{A}_{5}(CNT)=6{n}^{2}+\left(\frac{8\sqrt{42}}{13}+\frac{16\sqrt{10}}{13}+\frac{3\sqrt{7}}{4}-\frac{48\sqrt{2}}{17}-11\right)n-\left(\frac{20\sqrt{40}}{13}-\frac{4\sqrt{35}}{3}+\frac{16\sqrt{10}}{13}+\frac{3\sqrt{7}}{8}-\frac{16\sqrt{5}}{9}+\frac{48\sqrt{2}}{17}-5\right)$$

**Proof:** For $\,n\ge 3$, carbon nanotube graph has nine types of edges based on the sum of the degrees of neighborhood. This sort of edge partition given below in Table 4.

i. The fourth version of ABC index is defined as
  $$AB{C}_{4}(G)=\sum _{xy\in E(G)}\sqrt{\frac{{s}_{x}+{s}_{y}-2}{{s}_{x}{s}_{y}}}$$
  We construct the relation for $AB{C}_{4}$ index of carbon nanotube graph using Table 4, that is;
  $$AB{C}_{4}(CNT)=\frac{8}{3}{n}^{2}+\left(\frac{1}{2}\sqrt{\frac{7}{2}}+\sqrt{\frac{10}{3}}+\frac{22\sqrt{2}}{15}+\frac{2\sqrt{22}}{21}-\frac{14}{3}\right)n-\left(\frac{1}{2}\sqrt{\frac{7}{2}}+\sqrt{\frac{10}{3}}\,+\frac{\sqrt{2}}{3}-2\sqrt{\frac{7}{5}}+5\sqrt{\frac{22}{21}}-8\sqrt{\frac{2}{7}}+\frac{10}{9}\right)$$
ii. The fifth version of geometry index is defined as

$$G{A}_{5}(G)=\sum _{xy\in E(G)}\frac{2\sqrt{{s}_{x}{s}_{y}}}{{s}_{x}+{s}_{y}}$$

**Table 4:** Edge partition of CNT graph based on the sum of the degrees of neighborhood vertices.

(*s*_*x*_, *s*_*y*_)	Number of edges
(4, 5)	$$4$$
(5, 5)	2n
(5, 7)	$$8$$
(5, 8)	$$4(n-1)$$
(6, 7)	$$2(2n-5)$$
(7, 9)	$$2n-1$$
(8, 8)	$$2(n-1)$$
(8, 9)	$$4(n-1)$$
(9, 9)	$$6{n}^{2}-15n+7$$

Similarly, the $G{A}_{5}$ index of CNT graph calculated through the values of Table 4, and after easy simplification, the required index is;

$$G{A}_{5}(CNT)=6{n}^{2}+\left(\frac{8\sqrt{42}}{13}+\frac{16\sqrt{10}}{13}+\frac{3\sqrt{7}}{4}-\frac{48\sqrt{2}}{17}-11\right)n-\left(\frac{20\sqrt{40}}{13}-\frac{4\sqrt{35}}{3}\,+\frac{16\sqrt{10}}{13}+\frac{3\sqrt{7}}{8}-\frac{16\sqrt{5}}{9}+\frac{48\sqrt{2}}{17}-5\right)$$

**Preposition 1.1**. The $\,AB{C}_{4}$ and $G{A}_{5}\,indices$ of carbon nanotube graph for $n=2$ are;

$${\rm{i}}.\,AB{C}_{4}(CNT)=\frac{4}{9}+2\sqrt{\frac{7}{5}}+9\frac{\sqrt{2}}{5}+\sqrt{\frac{10}{3}}+\sqrt{\frac{22}{5}}+\frac{31}{2\sqrt{14}}$$

$${\rm{ii}}.\,G{A}_{5}(CNT)=5+\frac{48\sqrt{2}}{17}+\frac{16\sqrt{5}}{9}+\frac{9\sqrt{7}}{8}+\frac{16\sqrt{10}}{13}+\sqrt{35}$$

**Proof:** The carbon nanotube graph has eight types of edges based on the sum of the degrees of neighborhood. The partition of the edges, based on the degrees of the neighborhood, is shown in the following table.

i. The fourth version of ABC index is defined as
  $$AB{C}_{4}(G)=\sum _{xy\in E(G)}\sqrt{\frac{{s}_{x}+{s}_{y}-2}{{s}_{x}{s}_{y}}}$$
  Thus, the values of Table 5 and the above expression, gives the $AB{C}_{4}$ index of carbon nanotube graph.
  $$AB{C}_{4}(CNT)=\frac{4}{9}+2\sqrt{\frac{7}{5}}+9\frac{\sqrt{2}}{5}+\sqrt{\frac{10}{3}}+\sqrt{\frac{22}{5}}+\frac{31}{2\sqrt{14}}$$

**Table 5:** Edge partition of CNT graph based on sum of the degrees of neighborhood vertices for $\,n=2$.

(*s*_*x*_, *s*_*y*_)	Number of edges
(4, 5)	$$4$$
(5, 5)	$$2$$
(5, 7)	$$6$$
(5, 8)	$$4$$
(7, 9)	$$3$$
(8, 8)	$$2$$
(8, 9)	$$4$$
(9, 9)	1
ii. The fifth version of geometry index is defined as

$$G{A}_{5}(G)=\sum _{xy\in E(G)}\frac{2\sqrt{{s}_{x}{s}_{y}}}{{s}_{x}+{s}_{y}}$$

The $G{A}_{5}$ index of CNT graph evolved through Table 5 and above expression $G{A}_{5}(G)$. After few steps of straightforward computations, the required index is;

$$G{A}_{5}(CNT)=5+\frac{48\sqrt{2}}{17}+\frac{16\sqrt{5}}{9}+\frac{9\sqrt{7}}{8}+\frac{16\sqrt{10}}{13}+\sqrt{35}$$

## Results and Discussions

In this study, we developed the formulae for calculating the ABC, GA, $AB{C}_{4}$ and, $G{A}_{5}$ topological indices for the 2D structures of hexagonal boron nitride and carbon nanotubes. These results make a significant contribution to the investigation of chemical graph theory, quantum chemistry, QSPR, and QSAR. The results of the study are as follows: **Hexagonal boron nitride graph (*BN*)** $\forall \,n\ge 2$

$$ABC(BN)=\sqrt{3}{n}^{2}-4\left(\frac{1}{\sqrt{3}}+\sqrt{2}\right)n+\left(\frac{1}{\sqrt{3}}-5\sqrt{2}\right)$$

$$AB{C}_{4}(BN)=\frac{4}{3}{n}^{2}+4\left(\frac{\sqrt{2}}{3}+\frac{22}{21}-\frac{8}{9}\right)n+\left(2\sqrt{\frac{7}{5}}-8\sqrt{\frac{22}{21}}+8\sqrt{\frac{2}{7}}+\frac{20}{9}\right)$$

$$GA(BN)=3{n}^{2}-4\left(1-\frac{4\sqrt{6}}{7}\right)n+7$$

$$G{A}_{5}(BN)=3{n}^{2}+\left(\frac{16\sqrt{42}}{13}+\frac{3\sqrt{7}}{2}-8\right)n-\left(\frac{32\sqrt{42}}{13}-\frac{4\sqrt{35}}{3}+\frac{4\sqrt{7}}{2}-\frac{16\sqrt{5}}{9}-7\right)$$

**Carbon nanotubes Graph (** ${\boldsymbol{CNT}}$**)** ${\boldsymbol{\forall }}\,{\boldsymbol{n}}{\boldsymbol{\ge }}{\bf{2}}$

$$ABC(CNT)=4{n}^{2}+\left(5\sqrt{2}-\frac{14}{3}\right)n-\sqrt{2}$$

$$GA(CNT)=6{n}^{2}-\left(\frac{25-16\sqrt{6}}{5}\right)n+\left(4-\frac{12\sqrt{6}}{5}\right)$$

**Carbon nanotubes Graph** ${\boldsymbol{\forall }}\,{\boldsymbol{n}}{\boldsymbol{\ge }}{\bf{3}}$

$$AB{C}_{4}(CNT)=\frac{8}{3}{n}^{2}+\left(\frac{1}{2}\sqrt{\frac{7}{2}}+\sqrt{\frac{10}{3}}+\frac{22\sqrt{2}}{15}+\frac{2\sqrt{22}}{21}-\frac{14}{3}\right)n-\left(\frac{1}{2}\sqrt{\frac{7}{2}}+\sqrt{\frac{10}{3}}\,+\frac{\sqrt{2}}{3}-2\sqrt{\frac{7}{5}}+5\sqrt{\frac{22}{21}}-8\sqrt{\frac{2}{7}}+\frac{10}{9}\right)$$

$$G{A}_{5}(CNT)=6{n}^{2}+\left(\frac{8\sqrt{42}}{13}+\frac{16\sqrt{10}}{13}+\frac{3\sqrt{7}}{4}-\frac{48\sqrt{2}}{17}-11\right)n-\left(\frac{20\sqrt{40}}{13}-\frac{4\sqrt{35}}{3}\,+\frac{16\sqrt{10}}{13}+\frac{3\sqrt{7}}{8}-\frac{16\sqrt{5}}{9}+\frac{48\sqrt{2}}{17}-5\right)$$

For ${\boldsymbol{n}}=2$ the fourth version of atom-bond connectivity index, and fifth version of geometric-arithmetic index of carbon nanotube graph are.

$$\begin{array}{rcl}AB{C}_{4}(CNT) & = & \frac{4}{9}+2\sqrt{\frac{7}{5}}+9\frac{\sqrt{2}}{5}+\sqrt{\frac{10}{3}}+\sqrt{\frac{22}{5}}+\frac{31}{2\sqrt{14}}\\ G{A}_{5}(CNT) & = & 5+\frac{48\sqrt{2}}{17}+\frac{16\sqrt{5}}{9}+\frac{9\sqrt{7}}{8}+\frac{16\sqrt{10}}{13}+\sqrt{35}\end{array}$$
